# Mechanosensitive channel candidate MCA2 is involved in touch-induced root responses in *Arabidopsis*

**DOI:** 10.3389/fpls.2014.00421

**Published:** 2014-08-21

**Authors:** Masataka Nakano, Rika Samejima, Hidetoshi Iida

**Affiliations:** Department of Biology, Tokyo Gakugei University, Koganei-shiTokyo, Japan

**Keywords:** mechanosensitive channel, *Arabidopsis*, root, skewing, waving, calcium, touch response, mechanical stress

## Abstract

The Ca^2+^-permeable mechanosensitive (MS) channel is a mechanical stress sensor. We previously reported that *Arabidopsis* MCA1 and its paralog MCA2 functioned individually as Ca^2+^-permeable MS channels. In the present study, we showed that the primary roots of the *mca2*-null mutant behaved abnormally on the surface of hard medium. First, primary roots are known to exhibit a skewing growth pattern on the surface of vertically placed agar medium. On such surface, the primary roots of *mca2*-null skewed more than those of the wild type. Second, when seedlings were grown on a tilted agar surface, the primary root of *mca2*-null showed abnormal waving patterns. Third, wild-type seedlings eventually died when grown on horizontally placed 3.2% gelrite medium, which was too hard to allow the primary roots of the wild type to penetrate, because their primary roots sprang from the surface of the medium and may have been unable to absorb water and nutrients. In contrast, the primary roots of *mca2*-null, but not those of *mca1*-null, were able to creep over the surface of the medium and grow. Fourth, when grown on the surface of 3.2% agar medium supplemented with 30 mM CaCl_2_, only *mca2*-null grew with a root that coiled in a clockwise direction. Lastly, on the surface of vertically placed rectangular plates that allowed primary roots to grow vertically down to the frame of the plate, wild-type primary roots grew horizontally after touching the frame at an angle of 90^∘^. During the horizontal growth, only the extreme root tips maintained contact with the frame. In contrast, the primary roots of *mca2*-null allowed not only the extreme root tips, but also the meristem and elongation zones to maintain contact with the frame during horizontal growth. These results suggest that MCA2 is involved in touch-related root responses.

## INTRODUCTION

Plant roots can sense and respond to various physical and chemical environments. Mechanical stimulation or touch represents one such environment. Roots grow downward and parallel to the gravity vector. However, roots avoid obstacles in the soil by changing the direction of growth. Roots were found to grow with a deviation from the gravity vector under experimental conditions in which roots could grow on the surface of vertical hard agar medium. This deviation is referred to as skewing. It does not occur in roots grown embedded in agar. The direction of skewing is to the left in most *Arabidopsis* (*Arabidopsis thaliana*) ecotypes if roots are observed from the front of the agar plate (Rutherford and Masson, 1996). Another appearance of roots grown on vertical surface is waving, a sinusoidal wave-like growth pattern. These growth patterns may be affected by gravity, touch-induced root tip rotation (Okada and Shimura, 1990; Oliva and Dunand, 2007), and root-gel interaction (Thompson and Holbrook, 2004; Oliva and Dunand, 2007). Models to explain how roots skew and wave have already been reviewed (Oliva and Dunand, 2007; Roy and Bassham, 2014). Recent studies in space demonstrated that skewing and waving were gravity-independent (Paul et al., 2012; Roux, 2012).

Mutants showing abnormal phenotypes have been isolated to gain mechanistic insights into skewing and waving at the molecular level. The characterization of some of these mutants revealed that the following gene products are involved in skewing and/or waving: α- and β-tubulins (Thitamadee et al., 2002; Ishida et al., 2007) and the auxin transporters, AUX1 and PIN2 (Okada and Shimura, 1990). This characterization suggests that after sensing a touch with the surface of the plate, roots skew and/or wave by changing microtubule organization and differential auxin fluxes (reviewed in Oliva and Dunand, 2007; Roy and Bassham, 2014). However, the molecules responsible for sensing mechanical stimuli generated by root-surface interactions have not yet been identified.

MCA1 (locus: At4g35920) and its paralog MCA2 (locus: At2g17780) are Ca^2+^-permeable mechanosensitive channel candidates in *Arabidopsis* (Nakagawa et al., 2007; Yamanaka et al., 2010; Nakano et al., 2011; Furuichi et al., 2012; Shigematsu et al., 2014; reviewed in Kurusu et al., 2013). Both share 73% identity in their amino acid sequences, exhibit Ca^2+^ influx activities, and were expressed in all the organs examined, including roots, stems, leaves, flowers, and sliques, by Northern blotting or RT-PCR (Nakagawa et al., 2007; Yamanaka et al., 2010). Histochemical staining assays have shown that *MCA1-*promoter::*GUS* and *MCA2-*promoter::*GUS* are both expressed in the vascular tissues of cotyledons, leaves, and roots. In addition, horizontal sectioning of roots has shown that both gene constructs are expressed in the stele and endodermis, but not in the cortex or epidermis (Yamanaka et al., 2010). Neither *MCA1-*promoter::*GUS* nor *MCA2-*promoter::*GUS* is expressed in the columella or peripheral cap. Our published and unpublished studies demonstrated that MCA1 and MCA2 were responsible for an increase in [Ca^2+^]_cyt_ with a hypo-osmotic shock (Nakagawa et al., 2007).

In spite of these similarities, MCA1 and MCA2 have distinct functions and expression patterns *in planta*. MCA1, but not MCA2, is involved in root penetration into hard agar medium from soft agar medium (Nakagawa et al., 2007). The deletion of *MCA2*, but not *MCA1*, caused a detectable decrease in Ca^2+^ influx in roots (Yamanaka et al., 2010). Although *MCA1-*promoter::*GUS* is expressed in the promeristem and adjacent elongation zone of the roots, *MCA2-*promoter::*GUS* is not (Yamanaka et al., 2010).

In the present study, we showed that the primary roots of the *mca2*-null mutant, but not those of the *mca1*-null mutant, exhibited abnormal skewing and waving patterns and proposed that one of MCA2 functions may be to act as a mechanosensor to perceive root-gel interactions.

## MATERIALS AND METHODS

### PLANT MATERIALS AND GROWTH CONDITIONS

The Columbia-0 (Col-0) ecotype of *Arabidopsis* (*Arabidopsis thaliana*) and its isogenic, transgenic lines were used. The *mca1*-null, *mca2*-null, and *mca1*-null *mca2*-null mutant lines produced by the insertion of T-DNA was described previously (Nakagawa et al., 2007; Yamanaka et al., 2010). For the sake of conciseness, the word “null” was omitted hereafter.

Regarding complementation by the *MCA2* gene, the T-DNA clone pGreenII0229-MCA2 was used for plant transformation (Yamanaka et al., 2010). T3 homozygous lines were used to examine phenotypes.

*Arabidopsis* seeds were sterilized with 20% sodium hypochlorite solution (1% active chlorine) and 0.1% Triton X-100 for 10 min followed by five consecutive rinses in sterilized Milli-Q water. The seeds were stratified at 4^∘^C for 3 days in the dark and plated on half-strength Murashige and Skoog (1/2 MS) medium supplemented with 1% sucrose and an appropriate concentration of Bacto-agar (Becton, Dickinson and Company, NJ, USA) or gelrite (Wako Pure Chemical Industries, Ltd., Osaka, Japan). Seedlings were incubated in a growth chamber at 22^∘^C with 70–100 μmol s^-1^ m^-2^ fluorescent light in a photoperiod of 16 h light/8 h dark.

### ROOT SKEWING ASSAY

Seedlings were incubated on the surface of vertically oriented 1/2 MS medium containing 1% sucrose and either 1.6% agar or 0.8% gelrite. Alternatively, seedlings were incubated on the horizontal surface of 1/2 MS medium containing 1% sucrose and either 1.6% agar or 0.8% gelrite. 7 days after sowing, the primary roots of seedlings were photographed with a digital camera (Sony, DSC-Hx30V, Tokyo or Ricoh, CX5, Tokyo) from the front of the plates, and the angle of root skewing was measured quantitatively using ImageJ software.

### ROOT WAVING ASSAY

Seedlings were incubated on the tilted surface of 1/2 MS medium containing 1% sucrose and 1.6% agar. During this incubation, the plates were kept tilted 30^∘^ from vertical for the growth direction. 7 days after sowing, the primary roots of seedlings were photographed as above and analyzed for the number of waves per root, the amplitude of waves, and the wavelength using ImageJ software.

### CFR ASSAY

Seedlings were grown on the surface of vertically oriented 1/2 MS medium containing 1% sucrose and either 1.6% agar or 0.8% gelrite. Photographs of roots were taken 7 days after sowing with a digital camera (Leica DFC-300-FX, Wetzlar, Germany) under a stereomicroscope (Leica, M165FC).

### ROOT PENETRATION AND VIABILITY ASSAYS OF PLANTS GROWN ON IMPENETRABLE MEDIUM

Seedlings were grown on 1/2 MS medium containing 1% sucrose and 0.3, 0.8, 1.6, or 3.2% gelrite, and the ratio of penetrated primary roots to unpenetrated ones was quantified 7 days after sowing. Sideway views of the primary roots were photographed with a stereomicroscope (Leica, MZ12.5) 4 days after sowing. The ratio of the viability of seedling on 3.2% gelrite was quantified 14 days after sowing.

### COILING OF THE PRIMARY ROOT ON HARD AGAR MEDIUM WITH EXCESS SALTS

Seedlings were grown on 1/2 MS medium containing 1% sucrose and 3.2% agar, supplemented with various salts. The ratio of root penetration and coiling was quantified 7 days after sowing.

### MEASUREMENT OF GEL HARDNESS

The physical hardness of agar media with or without 30 mM CaCl_2_ was measured with a rheometer (Shimadzu, EZ Test, Kyoto).

### ROOT BENDING ASSAY

Seedlings were incubated on the surface of vertically oriented 1/2 MS medium containing 1% sucrose and 0.8% gelrite. Rectangular Petri dishes were used to let the root tips encounter the frame of the dishes at an angle of 90^∘^ several days after sowing. One day after the extreme root tips had reached the frame, photographs were taken with a digital camera (Canon, EOS40D, Tokyo) under a stereomicroscope (Leica, MZ12.5).

### STATISTICAL ANALYSIS

Statistical significance was determined using unpaired Student’s *t*-test, with a maximum *p* value of < 0.05 required for significance.

## RESULTS

### ABNORMAL ROOT SKEWING IN THE *mca2* MUTANT

The *mca1* mutant, but not the *mca2* mutant, was previously shown to be defective for root penetration into hard medium containing 1.6% agar from soft medium containing 0.8% agar (Nakagawa et al., 2007; Yamanaka et al., 2010). To further explore the root phenotypes of mutants lacking either *MCA1* or *MCA2* or both, we grew these mutants on the surface of agar plates placed vertically rather than horizontally. We first examined root skewing. 7 days after sowing on vertically placed 1.6% agar plates, the primary roots of the *mca1*, *mca2*, and *mca1 mca2* mutants as well as those of the Col-0 wild type were examined for skewing. **Figure 1A** shows that the primary root of the wild type skewed slightly leftwards with a wavy phenotype when viewed from the front of the plate. Similar behavior was observed in the *mca1* and *mca1 mca2* mutants. In contrast, the primary root of the *mca2* mutant skewed more to the left than that of the others. A quantitative analysis (**Figure 1C**) clearly confirmed the skewing phenotype of *mca2*. The leftward skewing-angle of approximately two-thirds of the *mca2* population was between 16 and 45^∘^, while that of the other mutants and the wild type was mainly between 0 and 15^∘^ (**Figure 1D**). A complementation line (*mca2/MCA2*) showed the wild-type phenotype, which indicated that the skewing phenotype could be attributed to deletion of the *MCA2* gene.

**FIGURE 1:** **The *mca2* mutant displayed abnormal root skewing phenotypes on vertical surfaces. (A,B)** Root skewing phenotypes. Seedlings of the *mca1*, *mca2*, and *mca1 mca2* mutants and the wild type were grown on the vertical surfaces of 1.6% agar **(A)** and 0.8% gelrite **(B)** plates. 7 days after sowing, photographs were taken and examined for quantitative analysis. Scale bars = 1.0 cm. **(C)** A schematic drawing of skewing-angle measurements. a, angle. When roots had warped during growth, the distal and proximal ends of the roots were connected by a straight line and the angle was measured with respect to the vertical line.** (D,E)** Root skewing angles on 1.6% agar and 0.8% gelrite plates, respectively. The frequencies (%) of the root skewing direction at intervals of 15^∘^ are represented by the length of the bars. Leftward and rightward directions are represented as a plus and minus, respectively.

Since root waving is affected by gelling polymers (Buer et al., 2006), we performed the same experiment as that above, except for the use of gelrite (0.8%) as a gelling polymer instead of agar. **Figures 1B,E** showed that the primary root of the wild type and the *mca1* and *mca1 mca2* mutants skewed slightly to the right when viewed from the front of the plate. This direction was opposite to that observed on the surface of agar. The rightward skewing-angle of approximately three-fourths of this population was between 0 and -15^∘^. On the other hand, the primary root of the *mca2* mutant skewed randomly in both directions; however, rightward skewing was predominant and exaggerated. **Figure 1B** also showed that the primary root of all the lines examined did not exhibit a waving phenotype on the gelrite surface.

Therefore, the skewing direction and waving behavior differed because of differences in the gelling polymers used, which suggested that root-surface interactions rather than gravity may be important for skewing and waving.

### THE *mca2* MUTANT HAD SKEWED ROOTS THAT EMBEDDED IN GELS

Primary roots grow almost straight and vertical if they are embedded in agar medium (Rutherford and Masson, 1996). However, we found that the primary root of *mca2* seedlings did not follow this rule. In the present study, seeds were sown on 0.8% agar plates that were placed horizontally and incubated for 4 days. **Figure 2A** shows that the primary roots of *mca1*, *mca1 mca2* and *mca2/MCA2* as well as that of the wild type essentially grew straight and vertical. In contrast, the primary root of *mca2* grew with a skewing phenotype. Quantitative data showed that 35% of *mca2* primary roots skewed, while no primary root of the four other lines did (**Figure 2B**). None of the five lines had a waving phenotype (**Figure 2A**). Essentially the same results were obtained when 0.3% gelrite was used as a gel instead of agar (**Figures 2C,D**).

**FIGURE 2:** **Primary roots of the *mca2* mutant skewed even when embedded in the gels. (A,C)** Root skewing phenotypes. Seedlings of the *mca1*, *mca2*, and *mca1 mca2* mutants and the complementation line (*mca2/MCA2*) as well as the wild type were grown on 0.8% agar **(A)** and 0.3% gelrite** (C)** plates that were placed horizontally. To show representative root behavior in the gels, they were cut out with a razor blade near the seedlings 4 days after sowing and the side view of the seedlings was photographed. Scale bars = 1.0 mm.** (B,D)** Frequency (%) of root skewing in 0.8% agar and 0.3% gelrite, respectively. To quantify the frequency of skewing, seedlings growing on the plates were photographed overhead 4 days after sowing. Skewed roots were defined as those that extended outside of the circle with a 2.5 mm radius whose central point was the bottom of the shoot. The frequency (%) of skewed roots was calculated by dividing the number of skewed roots by the total number of roots examined. The number of the roots examined is as follows: in **(B)**, WT, 60, *mca1*, 34; *mca2*, 62; *mca1 mca2*, 26; *mca2/MCA2*, 69. In **(D)**, WT, 68, *mca1*, 58; *mca2*, 62; *mca1 mca2*, 44; *mca2/MCA2*, 59. *p > 0.05, **p < 0.00001.

### THE *mca2* MUTANT EXHIBITED ABNORMAL ROOT WAVING ON THE TILTED AGAR SURFACE

To examine the root-waving patterns of the *mca* mutants, 1.6% agar plates tilted at 30^∘^ were employed because tilting stably induces waving (Okada and Shimura, 1990). 7 days after sowing on the tilted plate, the primary roots of the *mca* mutants as well as those of the wild type were analyzed for waving. **Figure 3** shows a representative photograph of waving patterns. The waving patterns of *mca2* were abnormal. The wave number per primary root was reduced to one-third and the amplitude and wavelength of the wave were increased by approximately two-fold. Quantitatively, the number of waves per primary root in this mutant was 2.6, amplitude 1.0 mm, and wavelength 4.5 mm (**Table 1**). In contrast, the number of waves per primary root was 6.8–7.5, amplitude 0.6 mm, and wavelength 2.3–2.5 mm in the wild type, the *mca1* and *mca1 mca2* mutants, and the *mca2/MCA2* complementation line. Thus, the function of MCA2 may be important for the formation of waves and the determination of waveforms.

**FIGURE 3:** **The *mca2* mutant displayed abnormal root waving phenotypes on tilted surfaces. (A)** A schematic drawing of a 1.6% agar plate tilted 30^∘^ from vertical.** (B)** A representative morphology of the primary roots of the *mca1*, *mca2*, *mca1 mca2* mutants and the wild type grown on the plate shown in **(A)**. Photograph was taken 7 days after sowing. Scale bar = 1.0 cm. **(C)** A schematic drawing for a quantitative assessment of waving properties, such as the number of waves per root, the amplitude (a) and the wavelength (b). See **Table 1** for the results.

**Table 1:** Waveform features of primary roots grown on tilted agar surface.

Genotype	Number of waves per root	Amplitude (mm)	Wavelength (mm)
Wild type (*n* = 25)	7.5 ± 1.6	0.6 ± 0.1	2.3 ± 0.5
*Mca1* (*n* = 24)	7.4 ± 1.4	0.6 ± 0.1	2.4 ± 0.5
*mca2* (*n* = 25)	2.6 ± 1.6*	1.0 ± 0.3*	4.5 ± 1.5*
*Mca1 mca2* (*n* = 23)	6.8 ± 1.3	0.6 ± 0.2	2.4 ± 0.5
*mca2/MCA2* (*n* = 25)	6.5 ± 1.2	0.6 ± 0.2	2.3 ± 0.4

The data presented here were based on the experimental results shown in **Figure 3**. *p < 0.05 (*mca2* vs. other lines).

### CELL FILE ROTATION APPEARED TO BE NORMAL IN THE PRIMARY ROOTS OF *mca* MUTANTS

Although epidermal cell file rotation (CFR) along the root was previously shown to be nonessential for root skewing and waving (Buer et al., 2006), the handedness of the CFR has frequently been correlated with the direction of skewing (Rutherford and Masson, 1996; Ishida et al., 2007). Therefore, we observed the CFR of the *mca* mutants and the wild type grown on the vertical surface of 1.6% agar and 0.8% gelrite plates. As shown in **Figure 4**, no detectable CFR was observed in all the lines examined irrespective of the sort of gelling polymers. Although the primary roots of the *mca* mutants and the wild type skewed to the left on the agar surface (**Figures 1A,D**) and the right on the gelrite surface (**Figures 1B,E**), the CFR was not detectable for the *mca* mutants or the wild type on both agar and gelrite surfaces. Furthermore, no significant difference was observed in the CFR between *mca2* and the other lines. Thus, the abnormal skewing phenotypes of *mca2* described in the above sections could not be attributed to the abnormal handedness of the CFR. A previous study reported that the primary root of wild-type Col-0 seedlings did not show skewing or waving on the surface of vertical agar plates (Rutherford and Masson, 1996).

**FIGURE 4:** **The epidermal CFR was normal in the primary roots of the *mca* mutants.** The *mca1*, *mca2*,* and mca1 mca2* mutants and the wild type were grown on the vertical surface of 1.6% agar **(A)** and 0.8% gelrite **(B)** plates. Photographs were taken 7 days after sowing. Scale bars = 0.1 mm.

### *mca2* SEEDLINGS SURVIVED ON IMPENETRABLE MEDIUM DUE TO THEIR CREEPING PRIMARY ROOT

To further explore the behavior of the primary roots of the *mca* mutants, we grew them on horizontally placed plates containing 0.3, 0.8, 1.6, or 3.2% gelrite. The standard concentration of gelrite needed to support plant cultivation is 0.3%. Root penetration into gelrite medium was examined 7 days after sowing. **Figure 5A** showed that the *mca1*, *mca2*, and *mca1 mca2* mutants as well as the wild type grew on 0.3, 0.8, and 1.6% gelrite plates, and no significant differences were observed in the growth of seedlings between the four lines. However, only *mca2* was able to grow on 3.2% gelrite medium, whereas the other three lines (**Figure 5A**, far right panel) and the *mca2/MCA2* complementation line (photographs not shown) could not. We then quantified the ratio of penetrated to unpenetrated roots and found that the ratio was similar between the five lines in every gelrite medium tested; only * mca2* had a significantly lower ratio at 0.8% gelrite (*p* < 0.05) than the other three lines. It should be noted that the primary root of the *mca2* seedling that grew on 3.2% gelrite (**Figure 5A**, far right panel) was incapable of penetrating the medium (**Figure 5B**). Even 14 days after sowing, *mca2* survived, grew larger (**Figures 5C,D**) and eventually blossomed (data not shown). Similar, but relatively less obvious results were obtained when 3.2% agar was used instead of 3.2% gelrite (see the next section).

**FIGURE 5:** **Roots of the *mca2* mutant crept over the surface of impenetrable medium and let the mutant survive.** The *mca1*, *mca2*,* and mca1 mca2* mutants and the wild type were grown on the horizontal medium containing different concentrations of gelrite. **(A)** Representative photographs were taken 7 days after sowing. Note that only the *mca2* seedlings were able to grow well on 3.2% gelrite medium. **(B)** Penetration ratio of the primary roots of various mutants grown on media with different concentrations of gelrite. The data for each line were taken 7 days after sowing. The penetration ratio (%) was defined as the number of penetrated roots per the total number of roots for each line. The number of the roots examined is as follows: WT, 163, *mca1*, 112; *mca2*, 126; *mca1 mca2*, 113; *mca2/MCA2*, 91. Values are the mean ±SD. *p < 0.05.** (C)** A representative photograph of plants grown for 14 days on 3.2% gelrite. Note that the roots of the *mca2* mutant crept over the surface of the medium. **(D)** Quantitative representation of viable plants grown for 14 days on 3.2% gelrite. The number of the plants examined is as follows: WT, 135, *mca1*, 78; *mca2*, 135; *mca1 mca2*, 75; *mca2/MCA2*, 125.

To search for the cause of the survival of *mca2*, we closely examined its primary roots. 4 days after sowing, the primary roots of *mca1*, *mca1 mca2*, *mca2/MCA2* and wild-type seedlings sprang from the surface of 3.2% gelrite (**Figure 6**). In contrast, the primary root of *mca2* crept over the surface of the medium. The majority of the *mca2*’ primary roots appeared to be in close contact with the surface. We speculates that creeping roots can obtain water and nutrients from the surface of the medium, whereas sprang roots cannot.

**FIGURE 6:** **Root behaviors of various mutants on the impenetrable medium.** The *mca1*, *mca2*, and *mca1 mca2* mutants and the complementation line (*mca2/MCA2*) as well as the wild type were grown for 4 days on the impenetrable, 3.2% gelrite medium and photographed. Scale bar = 1.0 mm.

### COMPLEMENTARY EFFECTS OF EXOGENOUSLY ADDED Ca^2+^ ON ROOT PENETRATION WERE SMALL IN *mca2* BECAUSE OF INDUCED ROOT COILING

Since MCA2 is involved in Ca^2+^ influx in the root (Yamanaka et al., 2010), the penetration defect of * mca2* roots seen on horizontal hard gelrite medium (**Figure 5**) may be rescued by exogenous Ca^2+^. To test this possibility, we added 30 mM CaCl_2_ to 3.2% agar medium instead of 3.2% gelrite medium. Agar was employed here because of difficulties in solidifying gelrite in the presence of high concentrations of ions. We grew the *mca1*, *mca2*, and *mca1 mca2* mutants and the wild type on horizontal plates containing 0.8 or 3.2% agar or 3.2% agar with 30 mM CaCl_2_. The standard concentration of agar needed to support plant cultivation is 0.8%, and was, thus, used as a control. 7 days after sowing, the growth of *mca2* seedlings looked normal on 3.2% agar, like that on 0.8% agar (**Figure 7A**), except that the primary roots did not penetrate 3.2% agar (**Figure 7B**). On the other hand, the growth of the other four lines was poor on 3.2% agar and their primary roots did not penetrate it.

**FIGURE 7:** **Ca^2+^ rescued *mca1, mca1 mca2* and wild-type roots, but not *mca2* roots, from the impenetrable state and induced root coiling in *mca2*. (A)** The *mca1*, *mca2*,* and mca1 mca2* mutants and the wild type were grown on horizontal medium containing 0.8% agar, 3.2% agar, or 3.2% agar with 30 mM CaCl_2_ and photographed 7 days after sowing. A relatively large number of roots of *mca1*, *mca1 mca2*, and wild-type seedlings were observed on the surface of the 3.2% agar plate (center panel) because the roots could not penetrate and crept over the agar. The addition of CaCl_2_ reduced this creeping behavior (right panel). **(B)** Quantitative representation of the root penetration phenotype described in **(A)**. The penetration ratio (%) was expressed as the number of penetrated roots per the total number of roots counted. The number of the roots examined is as follows: WT, 208, *mca1*, 196; *mca2*, 211; *mca1 mca2*, 207; *mca2/MCA2*, 68. Values are the mean ±SD. *p < 0.05. **(C)** Ca^2+^-induced root coiling in *mca2* seedlings on 3.2% agar containing 30 mM CaCl_2_. Scale bars = 1.0 mm.** (D)** Quantitative representation of the root coiling phenotype observed in **(C)**. The number of the roots examined is as follows: WT, 222, *mca1*, 167; *mca2*, 225; *mca1 mca2*, 156; *mca2/MCA2*, 110. The coiling ratio (%) was expressed as the number of coiled roots per the total number of roots counted. Values are the mean ± SD. The majority (77%) of the coiled roots were right-handed.

When 30 mM CaCl_2_ was supplemented to 3.2% agar, the growth of *mca1*, *mca1 mca2*, and wild-type seedlings recovered to a normal level that was similar to that of *mca2* seedlings (**Figure 7A**, right panel). This effect of Ca^2+^ may be partially attributed to the recovery of the penetrating abilities in *mca1*, *mca1 mca2*, *mca2/MCA2* and wild-type seedlings (**Figure 7B**). However, Ca^2+^ did not increase the penetrating ability of *mca2* seedlings, but induced coiling (**Figure 7C**). Approximately 77 ± 11% (*n* = 212) of the primary roots coiled in *mca2* (**Figure 7D**) and the direction of these coils was mostly clockwise (77 ± 9% of the total).

Among the salts tested, including 30 mM CaCl_2_, 30 mM MgCl_2_, 30 mM MgSO_4_, 50 mM NaCl, and 50 mM KCl, these effects were found to be CaCl_2_-specific (data not shown). In addition, increases in the penetration abilities of *mca1*, *mca1 mca2*, *mca2/MCA2* and wild-type roots were not due to the softening of agar due to the addition of CaCl_2_ because no significant difference was observed in solidity between 3.2% agar and 3.2% agar containing 30 mM CaCl_2_ (0.61 ± 0.01 and 0.62 ± 0.04 N/mm^2^, respectively; *p* > 0.05).

### ELONGATION ZONES OF *mca2* PRIMARY ROOTS WERE DEFECTIVE IN THE BENDING RESPONSE

A previous study reported that when primary roots that were growing vertically downward encountered a barrier placed perpendicular to the direction of growth, they formed a step-like structure with bends forming in the central elongation zone (CEZ) and then the distal elongation zone (DEZ; Massa and Gilroy, 2003). We here referred to this behavior as the bending response. In the present study, seeds were sown on vertical rectangular plates containing 0.8% gelrite medium to allow the primary roots to grow vertically down on the surface of the medium. We designed experimental conditions that allowed the root tips to encounter the frame of the rectangular Petri dish at an angle of 90^∘^ several days after sowing. As shown in **Figure 8A**, the primary roots of *mca1*, *mca1 mca2*, *mca2/MCA2*, and wild-type seedlings showed the bending response, whereas that of the *mca2* seedlings did not. The primary root of the *mca2* seedlings allowed not only its extreme root tip, but also the meristem and elongation zones to keep in close contact with the frame of the plate during horizontal growth.

**FIGURE 8:** **Roots of the *mca2* mutant did not show the bending response at the DEZ when encountered a barrier. (A)** Representative images of roots showing the bending response. Roots were allowed to grow on the vertical surface of 0.8% gelrite medium and encounter the frame of the rectangular Petri dish at an angle of 90^∘^ several days after sowing. Photographs were then taken. Scale bar = 1.0 mm. The arrows indicate the centers of the CEZ and DEZ, positions of which conform to those described by Massa and Gilroy (). **(B)** A schematic drawing for measuring the angle of a root tip. a, angle. **(C)** The angle of root tips. The number of the roots examined is as follows: WT, 8, *mca1*, 7; *mca2*, 11; *mca1 mca2*, 8; *mca2/MCA2*, 8. Values are the mean ±SD. *p < 0.0001 (*mca2 vs*. other lines).

We quantified root tip angles to the frame of the rectangular Petri dish, as shown in **Figure 8B**, and found that the root tip angle of *mca2* was greater than that of other four lines and that there is no difference in the angle between the four lines (**Figure 8C**).

## DISCUSSION

In the present study, we showed that MCA2 was involved in regulating skewing and waving in *Arabidopsis* primary roots. The primary root of the *mca2* mutant showed an abnormally strong skewing phenotype not only on the surface of vertical plates, but also in gels made of agar or gelrite (**Figures 1** and **2**). In addition, the primary root also showed an abnormal waving phenotype with a bigger amplitude and longer wavelength than the wild-type primary roots (**Figure 3** and **Table 1**). Since MCA2 has Ca^2+^-permeable mechanosensitive channel activity (reviewed in Kurusu et al., 2013), the results of the present study provide a new insight into the molecular mechanisms underlying sensing and responding to the touch of the primary root with the surface of hard media, eventually regulating skewing and waving. To unravel the molecular mechanisms involved, many mutations related to skewing and waving have been identified (reviewed in Oliva and Dunand, 2007), including those in the auxin eﬄux carrier (*agr1/wav6/eir1/pin2*), auxin influx transporter (*wav5/aux1*), 1-aminocyclopropane-1-carboxyylic acid synthase involved in ethylene synthesis (*ect1*), α-tubulin 6 (*lefty1*), and α-tubulin 4 (*lefty2;* Okada and Shimura, 1990; Thitamadee et al., 2002; Yuen et al., 2005). Models accounting for the cellular process leading to skewing and waving have been postulated based on the characterization of these and other mutants (Oliva and Dunand, 2007; Roy and Bassham, 2014). However, the mechanisms by which roots sense a touch with the surface of gels has yet to be elucidated in detail. We here propose that MCA2 may play a role in sensing a mechanical stimulus due to a root-gel interaction in order to generate the early cellular response necessary for regulating the skewing and waving behaviors of roots.

### IMPORTANCE OF MCA2 IN ROOT-GEL INTERACTIONS

The strong skewing phenotype of * mca2* roots could be attributed to two possible causes. One is that *mca2* roots have lost the normal ability to sense touch with gels and thereby have deregulated themselves to skew. The other is that *mca2* roots have partially lost the gravity-sensing ability such that they cannot undergo complete vertical growth and thereby skews. We recently found that *mca2* roots appeared to be somewhat defective in the gravitropic response: after *mca2* seedlings growing vertically were placed horizontally, the start of vertical growth of their roots was delayed in agar medium (Nakano and Iida, unpublished observation). At present, however, it is hard to distinguish between the two possibilities because touch stimulation modulates the gravitropic response (Massa and Gilroy, 2003). In the case of this observation, for example, the reason for the delay can be explained in two ways. One is that the delay is simply due to a partial defect of *mca2* roots in sensing gravity. The other is that the delay is a secondary effect of the loss of the normal ability of *mca2* roots to sense touch with agar.

Thus we have no decisive data to distinguish completely between the abovementioned two possible causes of the strong skewing phenotype of *mca2* roots. However, the result that *mca2* roots as well as *MCA2*^+^ roots skew to fixed directions depending on the sort of hard gels (**Figure 1**) favors the former possibility, i.e., the loss of touch sensing. If the loss of gravity-sensing is a major reason for the strong skewing of *mca2* roots, the direction of skewing would be at random irrespective of the sort of gels. However, *mca2* roots skew more to the left on agar surfaces and to the right on gelrite surfaces, and this is stronger in *mca2* roots than in *MCA2*^+^ roots. Consistent with this speculation, recent experiments conducted in spaceflight have indicated that gravity is unnecessary for skewing and waving (Paul et al., 2012; Roux, 2012). Therefore, we propose that MCA2 may be involved in touch-sensing to regulate root behaviors.

### IMPORTANCE OF MCA2 IN THE BENDING RESPONSE OF ROOTS

Under natural environments, roots must distinguish between soft and hard soils after touching them and select soft ones to grow into further or sometimes must penetrate hard soils by strengthening themselves. MCA2 may be involved in these processes. When the *mca* mutants and the wild type were grown on 3.2% gelrite and 3.2% agar medium, which were hard enough to prevent the penetration of wild-type roots, the root tips of * mca1*, *mca1 mca2* and *mca2/MCA2* seedlings as well as those of wild-type seedlings appeared to persistently try to penetrate the gels and eventually let the whole roots spring up above the gel surface, resulting in the death of the seedlings (**Figure 6**). In contrast, *mca2* seedlings were able to survive under the same growth conditions because not only their root tips, but also the entire region of the roots made contact with the gel surface. This contact may enable the seedlings to incorporate water and nutrients from medium. MCA2 may participate in sensing the hardness of the soil in order to allow the roots to change their strength in response to soil hardness.

Another phenotype of *mca2* roots is a defect in the bending response. When the root tips of *mca1*, *mca1 mca2*, *mca2/MCA2* and wild-type seedlings encountered a barrier at an angle of 90^∘^, they bended at the CEZ and DEZ, causing a step-like growth. However, *mca2* primary roots were incapable of this type of growth at the DEZ (**Figure 8**). Similar to the behavior observed on the surface of the hard media as discussed above, the entire region of the roots made contact with the barrier. In natural situations, MCA2 could participate in sensing the presence of rocks in the soil to allow the roots to properly change direction.

The bending response was previously investigated in some detail by Massa and Gilroy (2003). Since the portion of the direct contact site with barriers is the columella, they removed central columella cells using laser ablation and examined the responses. It was found that columella-ablated roots still exhibited the bending response, although they had a shallower angle than untreated roots at the DEZ. Similar findings were obtained with roots in which the peripheral cap cells or whole cap cells had been removed. These results suggest that although the root cap is involved in the bending response to a certain degree, other regions in the root are more important. In this context, it is worthwhile to note that *mca2* roots are totally defective in the bending response at the DEZ.

### WHERE DOES MCA2 SENSE TOUCH STIMULATION?

In our previous study, a side view of GUS-stained seedlings revealed that *MCA2*-promoter::*GUS* was expressed in all regions of the primary root, except for the root cap, the meristematic zone, and the DEZ (Yamanaka et al., 2010). This expression pattern appears not to favor MCA2 being involved in the perception of touch stimulation in the root because it is easy to conceive that, as an initial contact site, the root cap and its surrounding region should be the most important site responsible for touch-perception during root growth. However, considering both the staining pattern of *MCA2*-promoter::*GUS* and the phenotypes of *mca2* roots presented here, we speculate that the root cap and its surrounding region are not the only site required for touch-perception during root growth; the CEZ and/or its shootward region are also needed. Accordant with this speculation, the bending response discussed above has been induced in cap-less roots (Massa and Gilroy, 2003). Furthermore, unilaterally applied agar induces the curvature away from this substance in maize (*Zea mays*) roots lacking the root tip (Ishikawa and Evans, 1992).

A cross-sectional view of GUS-stained primary roots has revealed that *MCA2*-promoter::*GUS* is expressed in the endodermis and stele, but not in the epidermis or cortex (Yamanaka et al., 2010). This finding indicates that cells expressing MCA2 do not touch directly with gels, obstacles, and the soil; however, MCA2 is required for touch perception. Although we do not have any data to explain this superficial discrepancy, we speculate that the impact of touch between roots and substances is strong enough to be transmitted from the epidermis to the endodermis and stele.

### DISTINCT FUNCTIONS OF MCA1 AND MCA2

Although MCA1 and MCA2 share 73% amino acid sequence identity and some of their structural features are identical, their expression regions and functions are not necessarily identical (Yamanaka et al., 2010; Nakano et al., 2011). The functions of MCA1 and MCA2 in roots are distinct. The present study demonstrated that MCA2, but not MCA1, was involved in the regulation of skewing and waving as well as the bending response. It is of interest to note that although *mca2* roots are defective in this regulation and response, the primary roots of the *mca1 mca2* double mutant behaved normally, similar to *mca1* and wild-type roots. We do not currently know the reason for this, but speculate that if both genes are knocked out, its effect is strong enough to induce compensatory gene expression or protein activation to suppress the phenotypes of the * mca2* mutant. Another plausible explanation is that the expression of the phenotypes of the *mca2* mutant requires the function of MCA1. Further mechanistic studies are necessary in order to elucidate the phenotype of the double mutant. It should be noted that the level of *MCA1* transcripts is not changed in the *mca2* mutant, and *vice versa* (Yamanaka et al., 2010). Therefore, the phenotypes of the *mca2* mutant presented here are not attributed to any changes in *MCA1* transcript levels.

Another distinct function of MCA1 and MCA2 is root penetration from soft agar into hard agar. We previously reported that the primary roots of the *mca1* mutant, but not those of the *mca2* mutant, were unable to enter lower, hard medium (containing 1.6% agar) from upper, soft medium (containing 0.8% agar) using the two-phase agar method (Nakagawa et al., 2007; Yamanaka et al., 2010). In this experiment, seeds were sowed on the surface of the soft (0.8%) agar medium and the primary roots were allowed to reach the hard (1.6%) agar medium 5–7 days after sowing. Therefore, it should be noted that this inability of * mca1* primary roots in penetration was observed under the conditions different from those observed in the present study, in which seeds were sowed directly on hard medium containing 3.2% gelrite (**Figures 5** and **6**) and 3.2% agar (**Figure 7B**). Apart from the differences in gel concentration and the sort of gels used between the two experiments, *mca1* primary roots showed an interesting phenotype in the previous study (Nakagawa et al., 2007). We noted that *mca1* primary roots were able to penetrate hard (1.6% agar) medium when the seeds were sowed directly on this medium (Nakagawa et al., 2007). This suggests that conditioning of primary roots may be established while they grow through the soft (0.8%) agar phase. In other words, primary roots could adapt themselves to environments in an early stage after germination, and the acquired properties may not be changed quickly.

The distinct function of MCA1 and MCA2 is also observed in Ca^2+^ uptake activity. The roots of the *mca2* mutant had less Ca^2+^ uptake activity than those of the wild type, while those of the *mca1* mutant had no detectable defect in this activity (Yamanaka et al., 2010). The present study showed that Ca^2+^ supplementation had no effect on the penetration of *mca2* roots into hard (3.2%) agar medium only (**Figure 7B**). The reason for this could be the low Ca^2+^ uptake activity by *mca2* roots.

### THE *MCA2* LOCUS

The isolation and characterization of mutants are powerful methodologies used to uncover the molecular mechanisms underlying biological phenomena of interest. Another useful method is quantitative trait locus (QTL) mapping, which provides information on the genetic loci of interest, leading to identification of the functions of gene products. Vaughn and Masson (2011) conducted QTL mapping of root skewing on agar surfaces using a recombinant inbred line population created from *Arabidopsis* accessions Cape Verde Islands (Cvi) and Landsberg *erecta* (L*er*), both of which show diverse and specific root growth behaviors on hard surfaces. Based on the results of this analysis and microarray analysis, these researchers suggested that the most plausible loci responsible for the difference in skewing between the two accessions are located at a region on chromosome 2, especially between position 9.3 and 11.2 Mb. We noted that this region was closed to the *MCA2* locus (At2g17780), which is located at 7.7 Mb on chromosome 2 of the Columbia (Col-0) ecotype of *Arabidopsis* (Nakagawa et al., 2007). This region and its surrounding regions could be a site important for root behavior in *Arabidopsis*.

In summary, we showed that MCA2 regulated root skewing and waving as well as the bending response. MCA2 did not affect the CFR. We suggest that mechanical perception by MCA2 may be performed not at the root cap and its surrounding region, but at the CEZ and/or more shootward regions

## AUTHOR CONTRIBUTIONS

Hidetoshi Iida managed the project. Hidetoshi Iida and Masataka Nakano planed the research. Masataka Nakano performed most of the experiments. Rika Samejima performed the root-skewing experiment. Masataka Nakano and Hidetoshi Iida wrote the paper.

## Conflict of Interest Statement

The authors declare that the research was conducted in the absence of any commercial or financial relationships that could be construed as a potential conflict of interest.
